RETRACTED

# Application and Effectiveness of Big Data and Artificial Intelligence in the Construction of Nursing Sensitivity Quality Indicators

**DOI:** 10.1155/2021/2087876

**Published:** 2021-09-21

**Authors:** Aie Chen, Xiaozhen Jiang, Fen Lian, Jing Wu, Xiaohua Weng, Wen Li

**Affiliations:** Blood Purification Department, Lishui People's Hospital of Zhejiang Province, Lishhui Zhejiang, 323000, China

## Abstract

In order to explore the quality management efficiency of applying big data and artificial intelligence in nursing quality index, a method of building a nursing management platform integrating nursing indicators and nursing events is proposed. Based on the investigation of the application demand of nursing information system, the method achieves timely data sharing and transmission through WLAN technology and realizes nursing management monitoring, nursing quality index enquiry, and automatic statistical analysis under the vertical management mode of nursing. The results showed that 77 people (73%) thought the time decreased, 19 people (18%) thought the time was the same, and 9 people (7%) thought the time increased. In terms of intelligent application and big data of nursing information management system, there is a significant difference in nursing management efficiency before and after using nursing management information system (*P* < 0.001). The nursing management control platform is designed and applied, and the nursing quality control method and actual management process are improved, which is very good for strengthening nursing quality management. The overall optimization of the quality control process is realized, which helps to mobilize the initiative and enthusiasm of nursing staff and continuously improve the effectiveness of nursing management and nursing efficiency.

## 1. Introduction

With the development and progress of the society, people's demand for medical treatment has been upgraded from the treatment of diseases to the integration of medical care. Nursing quality evaluation is an objective indicator reflecting this demand and is the key link and important basis of nursing quality management [1]. Scientific, reasonable, unified, and standardized nursing quality indicators are the main tools for evaluating nursing quality, with the help of which nursing services can be evaluated and supervised throughout the whole process [2]. Correct and effective use and analysis of nursing quality index data can timely find out the problems existing in nursing quality and safety management and provide a basis for managers to make decisions. In the context of the era of big data, nursing information discipline, which organically combines nursing science, computer science, and information science, emerges at the historic moment [3]. Nursing informatics will identify and process the collected data to provide the basis and direction for managers to make decisions or behaviors. The nursing quality management information system refers to the nursing quality score mark. Input the data into the computer, establish the database, store the information with the computer, carry out statistical analysis, and output the nursing work quality of each department, so as to accurately evaluate the quality of nursing work, find defects, and promote the continuous improvement of nursing quality [4]. How to use big data and artificial intelligence to optimize the function of nursing quality management information system is a topic that needs to be actively explored and solved by nursing management personnel. Some hospitals in China have started to use the hospital information system (HIS) based on mobile network equipment and distributed software development to improve the working efficiency and service quality. The nursing department cooperates with software companies [5]. We design and apply the nursing quality management system with smart phone as the terminal and big data analysis and nursing quality control platform as the core, adopt the mode of pilot before rolling out, and apply it in all nursing units of the hospital; it has promoted the informatization construction of nursing quality management and achieved good results in shortening the time of nursing quality control, optimizing the flow of nursing quality control and strengthening the quality control and tracking management in the process of nursing service [6].

RETRACTED

Guleng et al. proposed to update the national nursing sensitive quality index database and identified 9 indicators, including 2 structural indicators: the ratio of specialized nurses to other nursing staff and the number of nursing hours per day of patients, 2 process indicators: nursing staff satisfaction and patient satisfaction with health education, and 5 outcome indicators: skin integrity care, falls, incidence of nosocomial urinary tract infection, patients' satisfaction with general nursing, and patients' satisfaction with pain management [7]. Through the development, testing, and implementation of the nursing sensitivity index database, Cz et al. effectively collected nursing staffing, patient flow adverse events, hand hygiene, and other management data, which can be used to measure nursing performance, evaluate patient prognosis, and determine the quality and safety of nursing practice. In order to improve the quality of nursing, the “web version of nursing quality evaluation and improvement system” was developed, and the nursing quality database included 260 nursing indicators [8]. Dey et al. integrated the traditional strategies of Walker and Avante based on the concept matrix of Holzemer's model of health care research results. Four structural indicators were finally determined: 24 h patient nursing hours and nurse staffing (personnel mix, skill mix, and personnel ratio), and four outcome indicators were determined: the incidence of pressure sores, the incidence of falls (injuries), hospital-acquired infections, and patient (family) nursing satisfaction [9]. By investigating six non-university teaching hospitals in different regions, Zhou established five nursing sensitivity quality indicators, including screening for mental disorders, observation of mental disorders, malnutrition, and standardized pain assessment for patients after surgery in the rehabilitation room and hospital units. Risk identification of patients in hospital can be realized to effectively measure the quality of nursing [10].

RETRACTED

On the basis of current research, a nursing management platform combining nursing indexes and nursing events was proposed. Based on the survey of application needs of nursing information system, the method achieves data sharing and transmission in time through WLAN technology and realizes nursing management monitoring, nursing quality index inquiry, and automatic statistical analysis under vertical nursing management mode. The experimental results showed that there was a significant difference in nursing management efficiency before and after artificial intelligence and big data were applied to nursing information management system (*P* < 0.001). The design and application of nursing management and control platform can comprehensively improve the nursing quality management and control methods and actual processes, which is very beneficial to strengthen nursing quality management. The overall optimization of quality control process will help to fully mobilize the initiative and enthusiasm of employees, and continuously improve the effectiveness of nursing management and nursing efficiency.

## 2. Application of Artificial Intelligence and Big Data

### 2.1. Establishing a Medical Care Quality Management System

In order to meet the application requirements of nursing information system, the nursing information system has timely data sharing and transmission with his database, big data platform, and medical information docking system through WLAN technology and realized the functions of nursing management monitoring, statistical analysis of nursing quality indicators, quality control, and automatic feedback under the vertical nursing management mode. The hospital has established a nursing informatization research and development team, which is composed of the director of nursing management, director of nursing department, some head nurses, nursing backbone, and engineers, and holds regular special meetings to jointly develop and improve system functions. The information flow of the nursing quality indicator information system is shown in Figure 1.

RETRACTED

Through the data cleaning and processing, the relevant data of nursing quality indicators are presented in the form of a variety of visual charts. Diversified charts show problems with quality of care from a variety of perspectives, so that weaknesses can be quickly identified and corrected to reduce the occurrence of quality of care problems. The “number of cases of event type and department” in adverse events is taken as an example for specific explanation. According to the selected year, quarter, month, and day, the number of cases of department of event type is presented in the form of data table and histogram. The types of reported events were presented in the form of pie chart, line chart, and Platonic chart, and the number of cases of event types and departments were compared in the form of year-on-year trend chart according to different conditions [11]. At the same time, the data of the content of adverse events were extracted, the fishbone diagram was drawn, and the major cause, medium cause, and minor cause were analyzed. In addition, the presentation of some data correlated the nurses involved in the indicators with the patients, and the responsibility was transferred to people to avoid the occurrence of buck passing. Nursing managers can use PDCA or failure mode and effect analysis (FMEA) management mode to manage nursing staff who present nursing quality problems and problems related to them from all angles and levels [12].

#### 2.1.1. The Application of Medical Care Quality Management System

- *System Login*. The computer of the nurse station can be equipped with medical and nursing quality management software, and all nurses can log in through the work number, which can facilitate the nurses to query the feedback information and nursing quality inspection information, and the steering group can also query the nursing management quality at any time.
- *Set Inspection Standards*. We improve the nursing quality information base and input the index items and quality standards to be monitored into the system, so as to form a more standardized and reasonable structured information, which is helpful for the inspection team to check, for example, in the nursing department, nursing data collection items have been added to the reporting system of bad nursing problems, such as the cause of patients' falls, treatment measures and the degree of injury, etc., and the system can automatically generate indexes such as the rate of patients' falls and the number of accidents.
- *Quality Control of Smart Phones*. Nursing quality monitoring personnel realize quality monitoring at the bedside of patients through smart phones and take the inspection standard as the control index to timely input, store, and report the existing nursing problems; if the submission is not completed in time, the system will send a reminder message. At present, the hospital has achieved bedside monitoring, such as nursing document management, ICU nursing quality, graded nursing, patient satisfaction, quality nursing quality control, and emergency nursing management. Comparison of the incidence (%) of falls/falls in the nursing safety management application information system is shown in Table 1. Comparison of the incidence of stress injury (%) of nursing safety management application information system is shown in Table 2.

RETRACTED

It is mainly composed of nursing sensitive index and clinical basic quality index, which is involved in the reporting, review, control, and tracking of nursing quality indicators. The system can automatically extract the relevant data of statistical query and decision analysis module, nursing adverse event reporting system, nursing electronic evaluation sheet, and other modules, realizing the function of systematic query, automatic statistics, analysis, and feedback of nursing indicators. The nursing department and quality control staff can check the indicators and quality control progress of the whole hospital and various departments at any time through the nursing management platform and the dashboard of the nursing management end of the medical letter smart phone. It is sensitive to the actual nursery-patient ratio, the incidence of falling and falling, and the incidence of unplanned extubation. For example, the incidence rate of unplanned extubation in the whole hospital in every quarter can be queried and analyzed.

As can be seen from Tables 1 and 2, after the trend chi-square test, there were significant differences in the incidence of fall/fall and stress injury in the four quarters (*P* < 0.05). Specifically, the incidence of falls/falls and stress injuries decreased significantly from the first quarter to the fourth quarter.

### 2.2. The Application Effect of Artificial Intelligence and Big Data in Medical Care Quality Management

Through the application of advanced technologies such as artificial intelligence and big data in medical care quality management, 79% of nursing staff said that the system greatly saves the time of nursing quality control, and nursing staff can realize the automatic generation of nursing quality management reports through the input of nursing quality management problems in the system, and automatic statistics of nursing problems can help save the statistical time of nursing management personnel, which can not only shorten the time of nursing quality control but also improve the efficiency of nursing [13]. This is shown in Table 3.

RETRACTED

As can be seen from Table 3, the comparative analysis of nursing management efficiency before and after the application of nursing management information system has significant difference (*P* < 0.001), which shows that the nursing management efficiency has been significantly improved after implementation.

The accuracy, completeness, and objective authenticity of traditional manual statistics are difficult to be guaranteed, which affects the management effect. The big data platform integrates the previously dispersed, isolated, and static information into complete, continuous, and shareable dynamic information, which improves the accuracy, objectivity, and continuity of nursing quality management. As long as the quality inspection data in the nursing quality management information system supported by the big data platform are timely input, the background can automatically and accurately calculate the scores, analyze the proportion of various problems, and realize the objective quantification of the quality index data. The system accurately analyzes the daily work quality of each nurse and checks the details that can be traced, so that the behavior of nursing staff can be more standardized, to ensure and improve the quality of nursing safety.

## 3. Experimental Analysis

The nursing quality management system based on big data and intelligent mobile realizes the timely sharing and transmission of data with his database, big data platform, and medical information docking system through WLAN technology, so as to realize the nursing management monitoring under the vertical nursing management mode. It has the functions of statistical analysis of nursing quality indicators, bedsides quality control and automatic feedback. The hospital can set up a nursing information R&D team, and the nursing director, nursing department director, some head nurses, nursing backbone, and engineers will regularly hold special meetings to jointly develop and improve the system functions. The whole hospital went online to use the new mobile nursing quality management information system.

The nursing quality management platform can be installed on the computer of the nurse station on each floor and the head nurse and the nurse's work mobile phone. Some nurses can log in to the platform using their work number to view the ward nursing quality and the feedback information of the nursing department. The nursing quality supervision and education group can also report the operation of the platform to the platform development company at any time, bring more quality standards and index items that need to be monitored into the system to improve the nursing quality standard information base.

RETRACTED

Analysis of hospital data after using the system is shown in Table 4; 73% of nurses believe that the use of the system can shorten the time consumption of nursing quality control. Nurses only need to input the complete quality control problems into the system. The system can automatically classify and count various reports and nursing problems in nursing quality management, which can effectively reduce the time used by nursing managers for input and statistics. At the same time, it can also inquire and supervise the nursing quality problems in real time, which greatly saves the time of nursing quality control and improves the work efficiency.

*Traditional Manual Statistics*. Accuracy, integrity, and objective authenticity are difficult to guarantee, affecting the management effect. The big data platform integrates the previously scattered, isolated, and static information into complete, continuous, and shareable dynamic information, which improves the accuracy, objectivity, and sustainability of nursing quality management. In the nursing quality management information system supported by big data platform, as long as all kinds of quality inspection data are timely input, the background can automatically and accurately calculate the scores, analyze the proportion of all kinds of problems, and achieve the objective quantification of quality index data. The quality of each nurse's daily work execution can be accurately counted, and the details can be traced back, so that the practice of nurses can be more standardized, and the safety and quality of nursing can be guaranteed and improved.

After the medical staff input the patient's basic information, cost information, and work performance into the system, the nurse can provide medical care for each disease through the task panel corresponding to the bed, so as to provide personalized and high-quality nursing services. It can meet the needs of patients, close the relationship between nurses and patients, real-time early warning and reminder, and reduce work omissions. The effective implementation of the nursing check system standardizes the behavior of nurse practitioners. Through synchronous ward rounds of medical care in the mobile medical system, the consistency of patient information obtained by medical care is improved, effective communication between medical care and patients is strengthened, the quality of medical care service is further improved, and patient satisfaction is enhanced.

RETRACTED

The nursing quality management platform can give full play to the automatic statistical analysis function of big data and realize the refinement of data management. The platform automatically summarizes the problems of each department according to the input results, analyzes the data according to the problem ratio, and feeds back the problems of each department by exporting word documents, so that the corresponding department can formulate improvement measures to improve the quality of nursing. Through the nursing quality management platform, medical staff can know the basic information, cost information, and work execution of patients at a glance. Through the corresponding task panel, the responsible nurse can provide personalized and high-quality nursing services to meet the needs of patients, close the relationship between nurses and patients, and real-time early warning information to reduce work omissions.

Information technology can not only improve the reliability and timeliness of data but also assist nursing decision making to avoid potential nursing risks, reduce the total length of patient hospitalization, reduce the total cost of patient hospitalization, and increase patient turnover and potential income, so as to achieve better quality nursing services. Through accurate statistical analysis of nursing quality monitoring content assisted by information technology, the complex data are organized and the redundant system is simplified, which provides support for the acquisition and storage of massive data and realizes the sharing of data across nursing units. It is helpful for nursing managers to quickly grasp the general situation of nursing quality, which is an important guarantee for the realization of modern medical construction.

This paper designs a nursing quality control platform by connecting big data with intelligent nursing information system and practices and improves the processes and methods of nursing quality control, so as to strengthen quality management, optimize quality control process, and improve work efficiency and management efficiency. However, there is still a lot of work to be done in the closed-loop management of the whole process of informatization of human, financial, and material resources and it is necessary to further improve the system function and improve the quality of nursing quality management.

## 4. Conclusions

In order to explore the quality management efficiency of applying big data and artificial intelligence in nursing quality indicators, a nursing management platform combining nursing indexes and nursing events was proposed. Based on the survey of application needs of nursing information system, the method achieves data sharing and transmission in time through WLAN technology and realizes nursing management monitoring, nursing quality index inquiry, and automatic statistical analysis under vertical nursing management mode. The experimental results show that there is a significant difference in nursing management efficiency before and after the application of artificial intelligence and big data in nursing management information management system (*P* < 0.001), which is very beneficial to comprehensively improve nursing quality control methods and actual processes and strengthen nursing quality management. It can realize the overall optimization of quality control process, help to mobilize the initiative and enthusiasm of nursing staff, and continuously improve the effectiveness of nursing management and nursing efficiency.

RETRACTED

At present, the users of regional APPS are gradually increasing, but relatively remote areas and underdeveloped rural areas do not know much about the convenience measures of apps. Therefore, these preferential measures should be extended to rural areas.

## Figures and Tables

**Figure 1:** Information flow of the nursing quality indicator information system.

**Table 1:** Comparison of the incidence (%) of falls/falls in nursing safety management application information system.

Quarterly		Number of cases occurring (example)	Number of inpatients (person)	Incidence	*x* ^2^	The *P* value
Public before	Q 1	5	8567	0.078	53.261	0.017

After the misfortune	Q 2	4	9856	0.0652
	Q 3	3	8632	0.0432
	Q 4	3	9765	0.0311

**Table 2:** Comparison of the incidence (%) of stress injury in nursing safety management application information system.

Quarterly		Number of cases occurring (example)	Number of inpatients (person)	Incidence	*x* ^2^	The *P* value
Public before	Q 1	5	8567	0.058	26.311	0.041

After the misfortune	Q 2	4	9856	0.0456
	Q 3	3	8632	0.0321
	Q 4	3	9765	0.0211

**Table 3:** Comparative analysis of nursing management efficiency before and after the application of information system (min/month, ±S).

Eyes	Bad care events	Number of nurses under control	
	Data collation and control accounting analysis	Sampling inspection data sorting and control accounting analysis	Introduction: computer data collation and control accounting analysis
Public before	9982.66 ± 15.26	9998.22 ± 33.78	9980.11 ± 16.08
After the misfortune	68.55 ± 1.01	64.33 ± 6.74	141.22 ± 9.01
*x* ^2^	1995.675	980.211	3272.343
The *P* value	<0.001	<0.001	<0.001

RETRACTED

**Table 4:** Comparison of analysis time of nursing quality problems input before and after using the nursing quality management information system by nurses.

Project	Number of people	Percentage
Time reduction	77	73
The time is equal	19	18
Time increases	9	7

## Data Availability

The data used to support the findings of this study are available from the corresponding author upon request.
